# Intelligent Diagnosis of Cervical Cancer Based on Data Mining Algorithm

This article has been retracted.

**DOI:** 10.1155/2021/7690902

**Published:** 2021-11-13

**Authors:** Lei Zhang, Yuanyuan Zhu, Yuchen Song, Yaqing Han, Danli Sun, Shanshan Qin, Yingchun Gao

**Affiliations:** Nanjing Med Univ, Affiliated Huaian Peoples Hosp 1, Dept Obstet & Gynecol, Huaian, 223300 Jiangsu, China

## Abstract

The intelligent diagnosis of cervical cancer by using a class of data mining algorithms has important practical significance. In particular, the useful information included in a significant quantity of medical data may not only discreetly boost the development of medical technology but also detect cervical cancer in the future. This paper improves the data mining algorithm and combines image recognition technology and data mining technology to extract and analyze image features. Moreover, this paper makes full use of the information contained in the image to realize the segmentation of the cervical cancer cell image, select the feature vector according to the characteristics of the cervical cancer cell, and use the statistical classification method to design the classifier. The test results show that the automatic recognition effect of this system is good, and it has a good auxiliary diagnosis effect. Therefore, it can be verified in clinical practice in the follow-up.

## 1. Introduction

Various kinds of malignant lesions may develop in different areas of the body, among the illnesses that pose a danger to people's lives. Cervical cancer is the fourth highest cause of death in women, and it is something that women have long been worried about and should not be disregarded. Cervical cancer therapy is generally determined by the patient's tumor stage. The early stages of cancer are treatable with surgery if detected early enough [1]. Radical surgery for cervical cancer coupled with radiation and chemotherapy is the sole option if the tumor has progressed to an advanced stage and most lymph nodes have been metastasized or invaded [2]. However, the majority of women who are diagnosed with breast cancer are already in the late stages of the disease. By determining the stage of a patient's cervical cancer, doctors can better anticipate the likelihood of recurrence and tailor treatment accordingly. As a result, predictive biomarkers are playing an increasingly significant role in determining prognosis [3].

With the rapid development of technology, our ultimate goal is to mine the information contained within the data. The application fields of related data mining algorithms for processing big data are very wide, including different fields such as medical treatment, medicine, business activities, science, and social practice networks. This has a lot to do with what we do on a daily basis. To be sure, data mining algorithms that analyze large amounts of big data are intertwined with everything from online appointment registration in hospitals to intelligent illness diagnosis to traffic congestion management and catastrophe prediction. In addition to the enormous quantity, diversity of kinds, and fast updating, these data also represent the value that may be reaped from the data itself.

Data mining has slowly built up theoretical expertise over decades, such as classification and grouping. Among data mining's main areas of study, the classification issue entails creating a classification model using associated algorithms to evaluate and forecast categories of unknowns. Data sample attributes are used as inputs, and the category in which a data sample is classified is returned as an output. The categorization issue is a fictitious one created to distract attention from real-world issues. Cervical cancer mortality and morbidity rates are rising fast throughout the world, and the causes for this are many. While on the one hand reflecting the issue of an ageing population, it also represents some of the most important cancer risk factors. As an alternative, a growing number of nations are experiencing fast population growth and an ageing population, with cancer emerging as the leading cause of death. As the number of patients is increasing year by year, the complexity of cervical cancer lesions and the many uncertainties of suffering from cervical cancer and other factors have led to their clinical data showing a large number of clinical data, diversified data types, extremely fast development, and implicit features of high information value. Patients may be reluctant to provide some private information in relation to clinical data, resulting in the lack of specific clinical data; in other cases, the obtained clinical data contains noise and complex information. The abovementioned issues may be resolved by using conventional techniques. The restrictions are very severe, and the final result of solving the problem is not ideal. Therefore, the use of a type of data mining algorithm for the intelligent diagnosis of cervical cancer has important practical significance, especially the valuable information contained in a large amount of medical data cancer diagnosis promotes.

## 2. Related Work

Multiple logistic regression was used in the literature to determine the relationship between late diagnosis and Medicaid status before the disease was even identified [4]. The research examines whether Medicaid recipients are more likely than women who have not participated to be diagnosed with advanced cervical cancer. According to the findings, advanced illness was seen in 51% of Medicaid recipients and 42% of non-Medicaid recipients. Women from lower socioeconomic backgrounds and the elderly are more vulnerable. According to the data shown above, in order to guarantee that at-risk women get screening services, greater awareness is required [5]. There are about 370,000 new instances of cervical cancer each year, according to the research [6]. This accounts for approximately 10% of all new cases of cancer in the world. The first step in combating global cancer is to gather as much data as possible on its prevalence and death. Recent worldwide statistics [7] show that outcomes are comparable to those from 10 years ago, although there is some fluctuation in the figures. Regular and prompt examination inspection and treatment are very important. At the molecular level, the literature [8] studied the pathogenesis of cervical cancer through the implicit data of gene chips, explored malignant tumor markers, and provided a powerful solution for tumor prevention and treatment. The literature [9] investigated the practical usefulness of transvaginal real-time ultrasound elastography technology in the detection of cervical cancer. The combined use of tumor markers was addressed in the literature [10] for the diagnosis of cervical cancer. The effects of particular anti-HPV16E6 ribozymes on cervical cancer cell phenotypic and gene expression have been addressed in the literature [11].

As we all know, for women over 30 years of age, this is the best choice for average risk [12]. The literature [13] evaluates the practices of primary care providers, stimulus factors, barriers to the use of common testing methods, and prolonged screening intervals for low-income women. Few of the patients provided in the literature [14] performed the combined test of the two screening methods, and it is recommended to extend the time interval appropriately. Among them, the excessively frequent screening and the error caused by the misreporting harm are all within the budget allowable range, thereby balancing the obstacles caused by extending the screening interval. Cervical cancer, the second-most incidence of female malignant tumors, is estimated by the World Health Organization. The probability that cancer is the first or second cause of death before the age of 70 is about 52.91%, and it is the third cause of death. The probability of four is about 12.79%. Finally, the remaining 59 countries (172 countries in total) rank cancer as the fifth to tenth [15]. The literature [16] proposed a detection method for diagnosing cervical cancer in women or identifying women who are sensitive to cervical cancer. By detecting Brn-3amRNA or Brn-3a protein (quality) in Brn-3a cells, it can then test whether women are sick or not or sensitive to it. Endometrial cancer and ovarian cancer were studied in genome-wide association research [17] to determine the features of the data composition. The literature [18] examines the diagnosis of ICC every six years in women with human immunodeficiency virus in order to determine the frequency of cervical cancer and compare it to women who are not infected with HIV. Women were the focus of a research performed in August. The research looked at whether or not the Pap test was infected with HIV.

## 3. Improved Application of Data Mining Algorithm in Intelligent Diagnosis of Cervical Cancer

The proportional difference model is often used in survival data where the mortality of different groups of patients converges over time. If it is assumed that there are two existing patient treatment groups (*i* = 1) and control groups (*i* = 2), the PO model assumes that the difference ratio between these two groups is a constant *c*:

(1) $$\begin{array}{c} \frac{F_{1}\left(t\right)/\left(1-F_{1}\left(t\right)\right)}{F_{2}\left(t\right)/\left(1-F_{2}\left(t\right)\right)}=c. \end{array}$$

Among them, *F*_1_(*t*) represents the cumulative distribution function of the treatment group, and *F*_2_(*t*) represents the cumulative distribution function of the control group. This model can be extended: we set *x* to represent the *p*-dimensional covariate vector and assume that the relationship between the constant *c* and the covariate is *c* = exp(*β*′*x*). Among them, *β* is the *p*-dimensional coefficient corresponding to the covariate. Therefore, until time *t*, the following relationship holds between the difference in the case of covariate *x* ≠ 0 and the difference in the case of covariate *x* = 0:

(2) $$\begin{array}{c} \frac{F\left(t\;|\;x\right)}{1-F\left(t\;|\;x\right)}=\frac{F_{0}\left(t\right)}{1-F_{0}\left(t\right)}\exp\left(\beta^{\prime }x\right). \end{array}$$

Among them, *F*(*t* | *x*) and *F*_0_(*t*), respectively, represent the unknown cumulative distribution function and the benchmark cumulative distribution function related to the failure time when the covariate *x* ≠ 0 and the covariate *x* = 0. Formula (2) can also be equivalently written in the following form [19]:

(3) $$\begin{array}{c} \log\text{it}\left\{\left[F\left(t\;|\;x\right)\right]\right\}=\wedge_{0}\left(t\right)+\beta^{\prime }x. \end{array}$$

Among them, ∧_0_(*t*) = log{*F*_0_(*t*)/(1 − *F*_0_(*t*))} represents the benchmark logarithmic difference function up to time *t*, which is the nonparametric function part to be approximated by Bernstein polynomials in this article. It is easy to know from its expression: ∧_0_(*t*) is monotonous and nondecreasing with respect to *t*, and there is ∧_0_(*t*) = −∞ and ∧_0_(*t*) = ∞. The proportional difference model has a reasonable biological explanation: the *j*th element *β*_*j*_ in the coefficient vector *β* can be interpreted as the unit contribution of the *j*th covariate to the logarithmic difference in failure time until time *t*. The biggest advantage of the score (logit> connection function is that the constant difference rate can be obtained from the model. For example, there are two different individuals, and the covariates are *x*_1_ and *x*_2_, respectively. From (3), it can be seen that the following expression holds:

(4) $$\begin{array}{c} \log\left\{\frac{F\left(t\;|\;x_{1}\right)/\left(1-F\left(t\;|\;x_{1}\right)\right)}{F\left(t\;|\;x_{2}\right)/\left(1-F\left(t\;|\;x_{2}\right)\right)}\right\}=\beta^{\prime }\left(x_{2}-x_{1}\right). \end{array}$$

This means that if the covariates between two individuals differ by one unit, then their logarithmic difference ratios differ by coefficient *β*, which can also be used as a further explanation for equation (3).

In addition, here, we point out the relationship between the logarithmic difference model and logistic regression, which is convenient for the calculation using the normal data enhancement method in the following text. Formula (2) can also be rewritten as follows:

(5) $$\begin{array}{c} F\left(t\;|\;x\right)=G\left(\wedge_{0}\left(t\right)+\beta^{\prime }x\right). \end{array}$$

Here, *G* represents the cumulative distribution function of the standard logistic random variable.

Unlike the Cox proportional hazard (PH) model, the PO model must estimate the nonparametric function Ao(*t*) while estimating the parameter *β*, which makes the parameter estimation problem under the PO model very complicated.

This theorem is at the heart of Bayesian analysis. The posterior probability of an occurrence is described by Bayes' theorem based on a priori information. Let us say we know that age has anything to do with the incidence of a certain malignancy, the factor of age can help people more accurately determine the probability of a person having cancer, that is, the role of prior information. The mathematical expression of Bayes' theorem is

(6) $$\begin{array}{c} P\left(A\;|\;B\right)=\frac{P\left(B\;|\;A\right)P\left(A\right)}{P\left(B\right)}. \end{array}$$

Among them, *A* and *B* both represent events, and the probability of occurrence of event *B* is *P*(*B*) ≠ 0. *P*(*A*\*B*) represents the conditional probability of event *A* occurring under the condition of event *B*, and *P*(*B*\*A*) represents the conditional probability of event *B* occurring under the condition of event *A*. *P*(*A*) and *P*(*B*) are the probability of event *A* and event *B* occurring independently, also called conditional probability.

Bayesian inference is based on Bayes' theorem. This method updates the posterior probability distribution of the parameters based on the prior probability and therefore incorporates both the prior hypothesis and a random sample to better serve the goal of statistical inference. More specifically, we use *π*(*θ*) to denote the prior distribution of the parameter *θ* of interest. The prior distribution of parameters can be any distribution in the parameter space, usually given by experience. *W* represents the observed sample, so the posterior distribution of parameter *θ* is the distribution of *θ* = *f*(*w* | *θ*)*π*(*θ*) under the conditions given by sample *W* = *w*, denoted as *π*(*θ* | *w*). For the case of the continuity density function, the density function formula of posterior distribution is [20]:

(7) $$\begin{array}{c} \pi \left(\theta \;|\;w\right)=\frac{h\left(w,\theta \right)}{m\left(w\right)}=\frac{f\left(w\;|\;\theta \right)\pi \left(\theta \right)}{\int_{\Theta }f\left(w\;|\;\theta \right)\pi \left(\theta \right)d\theta }. \end{array}$$

Among them, *h*(*w*, *θ*) = *f*(*w* | *θ*)*π*(*θ*) is the joint distribution of *w* and *θ*, and there is

(8) $$\begin{array}{c} m\left(w\right)=\int_{\Theta }f\left(w\;|\;\theta \right)\pi \left(\theta \right)d\theta , \end{array}$$

which is the marginal distribution of sample *w*. The posterior distribution function calculated in formula (7) combines the information given by the population (that is, the density function *f*), the sample and the prior. From the Bayesian point of view, all statistical inferences should be derived from the posterior distribution function *π*(*θ* | *w*), such as calculating the mean value and confidence interval of the parameters.

Model (2) is combined, and the likelihood function expression based on right-censored data is

(9) $$\begin{array}{c} L=\overset{n}{\underset{i=1}{\prod }}F{\left(R_{i}\;|\;x_{i}\right)}^{\delta_{i1}}{\left[F\left(R_{i}\;|\;x_{i}\right)-F\left(L_{i}\;|\;x_{i}\right)\right]}^{\delta_{i2}}{\left[1-F\left(L_{i}\;|\;x_{i}\right)\right]}^{\delta_{i3}}. \end{array}$$

Among them, *δ*_*i*1_, *δ*_*i*2_, and *δ*_*i*3_ are all indicative functions. When the value is 1, it means that the *i*th individual is left censored, right censored, and interval censored and satisfies *δ*_*i*1_ + *δ*_*i*2_ + *δ*_*i*3_ = 1.

This article defines the *i*th individual:

(10) $$\begin{array}{c} t_{i}=R_{i}I_{\left(\delta_{i1=1}\right)}+L_{i}I_{\left(\delta_{i1=0}\right)}. \end{array}$$

Therefore, based on the relationship between the PO model and logistic regression described in equation (5), this paper uses the following data enhancement methods:

(11) $$\begin{array}{c} z_{i}=\wedge_{0}\left(t_{i}\right)+\beta^{\prime }x_{i}+\in_{i},\;z_{i}\in C_{i},\\ \in_{i}∼N\left(0,\lambda_{i}\right),\lambda_{i}={\left(2\psi \right)}^{2},\psi_{1}∼\text{KS}. \end{array}$$

Among them, KS represents the distribution function of Kolmogorov-Smirnov distribution, and the specific expression is

(12) $$\begin{array}{c} \text{KS}\left(x\right)=1-2\overset{\infty }{\underset{j=1}{\sum }}{\left(-1\right)}^{j}e^{-2j^{2}x^{2}},\;x>0. \end{array}$$

Corresponding to formula (9), if there is *δ*_*i*1_ = 1, then there is *C*_*i*_ = (0, ∞). If there is *δ*_*i*2_ = 1, then there is *C*_*i*_ = (∧_0_(*L*_*i*_) − ∧_0_(*R*_*i*_), 0). If there is *δ*_*i*3_ = 1, then there is *C*_*i*_ = (−∞, 0). In the above data enhancement method, the logistic distribution of ∈_*i*_ can be derived from the scale normal mixed distribution with the Kolmogorov-Smirnov distribution. Therefore, under the transformation of formula (11), the likelihood function in formula (9) can be rewritten as [21]

(13) $$\begin{array}{c} L=\overset{n}{\underset{i=1}{\prod }}N{\left(z\right.}_{i};\wedge_{0}\left(t_{i}\right)+\beta^{\prime }x_{i}\lambda_{i}{\left\{I_{\left(z_{i}>0\right)}\right\}}^{\delta_{i1}}{\left\{I_{\left(\wedge_{0}\left(L_{i}\right)-\wedge_{0}\left(R_{i}\right)<z_{i}<0\right)}\right\}}^{\delta_{i2}}{\left\{I_{\left(z_{i}<0\right)}\right\}}^{\delta i3}\pi \left(\lambda_{i}\right). \end{array}$$

Among them, there is

(14) $$\begin{array}{c} \pi \left(\lambda_{i}\right)={\lambda_{i}}^{-1/2}\frac{KS\left(\lambda_{i}^{1/2}/2\right)}{4}. \end{array}$$

The main part of the above enhanced likelihood function expression (13) is the product of the constrained normal density, which is very beneficial to the Gibbs sampling method given below.

This article defines all parameters a priori in order to enhance the Bayesian approach by ensuring that the parameters not only offer adequate modeling flexibility but also enable efficient posterior computations. More specifically, this article specifies a multivariate normal prior *N*(*β*_0_, ∑_0_) for the regression parameter *β*, a normal prior *N*(*m*_0_, *v*_0_^−1^) for the coefficient *γ*_0_ of the Bernstein approximation polynomial, and an independent exponential prior Exp(*η*) for the remaining Bernstein coefficients *γ*_*i*_(*i* = 1, ⋯, *N*). Exponential priors can shrink relatively small coefficients to zero and thus can play a role in penalizing nonzero coefficients. In order to ensure sufficient modeling flexibility at the same time, this paper specifies a gamma super prior Ga(*a*_*η*_, *b*_*η*_) for the parameter *η*.

The initial values of all parameters are sampled from their prior distributions. The iterative steps of Gibbs sampling in this paper are as follows:

(1) For *i* = 1, ⋯, *n*, the algorithm extracts the latent variable *z*_*i*_.
  - If there is *δ*_*i*1_ = 1, the algorithm extracts samples of *z*_*i*_ from *N*(∧_0_(*t*_*i*_) + *β*′*x*_*i*_, *λ*_*i*_)*I*_(*z*_*i*_ > 0)_
  - If there is *δ*_*i*2_ = 1, the algorithm extracts samples of *z*_*i*_ from*N*(∧_0_(*t*_*i*_) + *β*′*x*_*i*_, *λ*_*i*_)*I*_(∧_0_(*L*_*i*_) − ∧_0_(*R*_*i*_) < *z*_*i*_ < 0)_
  - If there is *δ*_*i*3_ = 1, the algorithm extracts samples of *z*_*i*_ from *N*(∧_0_(*t*_*i*_) + *β*′*x*_*i*_, *λ*_*i*_)*I*_(*z*_*i*_ > 0)_
(2) The algorithm extracts samples of *γ*_0_ from the normal distribution *N*(*E*_0_, *W*_0_^−1^); among them, there is

(15) $$\begin{array}{c} W_{0}=v_{0}+\overset{n}{\underset{i=1}{\sum }}\lambda_{i}^{-1},\\ E=W_{0}^{-1}\left[v_{0}m_{0}+\overset{n}{\underset{i=1}{\sum }}\lambda_{i}^{-1}\left\{z_{i}-\overset{N}{\underset{k=1}{\sum }}\gamma_{k}b_{k}\left(t_{i},N\right)-\beta^{\prime }x\right\}\right]. \end{array}$$

For *k* = 1, ⋯, *N*, the algorithm draws samples of *γ*_*k*_. We set *W*_*k*_ = ∑_*i*=1_^*n*^*λ*_*i*_^−1^*b*_*k*_^2^(*t*_*i*_, *N*). If there is *W*_*k*_ = 0, the algorithm extracts *γ*_*k*_ from Exp(*η*); otherwise, the algorithm extracts *γ*_*k*_ from *N*(*E*_0_, *W*_*k*_^−1^)*I*_(*y*_*k*_ > *d*_*k*_^∗^)_. Among them, there is

(16) $$\begin{array}{c} E_{k}=W_{k}^{-1}\left[\overset{n}{\underset{i=1}{\sum }}\lambda_{i}^{-1}b_{k}\left(t_{i}\right)\left\{z_{i}-\gamma_{0}-\underset{k\prime \neq k}{\sum }\gamma_{k\prime }b_{k\prime }\left(t_{i}\right)-\beta^{\prime }x_{i}\right\}-\eta \right],\\ d_{k}^{*}=\max\left(c_{k}^{*},0\right),\\ c_{k}^{*}=\underset{i:\delta_{12}=1}{\max}\left[\frac{-z_{i}-\sum_{k\prime \neq k}\gamma_{k\prime }\left\{b_{k\prime }\left(R_{i}\right)-b_{k\prime }\left(L_{i}\right)\right\}}{b_{k}\left(R_{i}\right)-b_{k}\left(L_{i}\right)}\right]. \end{array}$$

The algorithm samples *β* from the normal distribution $N\left(\tilde{\beta },\tilde{\sum }\right)$; among them, there is

(17) $$\begin{array}{c} \sum^{\sim }={\left(\overset{-1}{\underset{0}{\sum }}+\overset{n}{\underset{i=1}{\sum }}\lambda_{i}x_{i}x_{i}^{\prime }\right)}^{-1},\\ \tilde{\beta }=\sum^{\sim }\left\{\overset{-1}{\underset{0}{\sum }}\beta_{0}+\overset{n}{\underset{i=1}{\sum }}\lambda_{i}^{-1}\left(z_{i}-\wedge \left(t_{i}\right)\right)x_{i}\right\}. \end{array}$$

The rejection sampling algorithm *l* is used to sample each *λ*_*i*_, and the fully conditional distribution of *λ*_*i*_ is proportional to the following formula:

(18) $$\begin{array}{c} \lambda_{i}^{-1/2}\exp\left\{-\frac{\lambda_{i}^{-1}}{2}{\left(z_{i}-\wedge \left(t_{i}\right)-\beta^{\prime }{\text{x}}_{i}\right)}^{2}\right\}\pi \left(\lambda_{i}\right). \end{array}$$

The algorithm samples *η* from distribution Ga(*a*_*η*_ + *k*, *b*_*η*_ + ∑_*k*=1_^*N*^*γ*_*k*_).

## 4. Intelligent Diagnosis of Cervical Cancer Based on Data Mining

When traditional data analysis methods deal with similar data, the effect is not ideal, and sometimes, even a lot of information contained in the data is lost, so that the inherent information and laws of the data cannot be mined. As a result, it is critical to understand the data processing and classification processes, as well as to extract the information hidden in the sample data.  Figure 1 depicts the processing of the cervical cancer classification issue in this paper.

Discretization of continuous attributes is the second step of data processing in this article. The basic process is shown in Figure 2.

The simplest discretization algorithm-binning technique is utilised in this article. Equal frequency binning and equal width binning are two common binning methods. Unsupervised discretization is used in the binning technique. There are many bins created when sorting an attribute data set from top to bottom. The technique of detection has nothing to do with the procedure. It is possible to get an equal-width binned dataset by using the equal-width binning technique, which uses a fixed width for each bin. To split the data into equal-sized boxes, use the equal-frequency box division technique.

The cervical cancer cell image automatic analysis system can be represented by the frame structure shown in Figure 3.

Image registration is mainly performed before other image processing steps. For example, it observes and compares satellite remote sensing images and medical images obtained under different modalities after registration. In addition, for example, it can obtain the topographic map of the vast land, or observe the lesion area of the medical image more conveniently, and register and fuse the CT and MRI images. One image is designated as a reference image, while the other as a floating image, when two pictures need to be registered. To accomplish the objective of matching the coordinates of the reference picture, the latter must employ a comparable transformation model. The first transformation model is generated based on the difference between the two pictures, and the initial transformation image and the reference image are compared for similarity. As long as the anticipated criteria are not being fulfilled, optimization algorithms are used to fine-tune the transformation model parameters. This procedure is repeated until the similarity measure falls within an acceptable range, at which point the registration process is complete. The differences between pictures of various modalities are primarily a limited range of translation and rotation, according to the features of the images in this article. Since Figure 4 shows how to determine a stiff transformation model, let us get into it.

The bilinear interpolation method uses the gray levels of the four neighboring pixels of the pixel to be found to perform linear interpolation in two directions, as shown in Figure 5.

For the removal of shadow areas, this paper considers the classification of colors based on HSI and Lab space, so white light image samples need to be added to participate in diagnosis. The specific algorithm flow is shown in Figure 6.

On the basis of the above research, the intelligent algorithm of this paper is used to verify the performance. Feature extraction is based on a certain pixel, pixel area, or specific target area as a unit and extracts a certain type of characteristic shown by the gray value of the area, usually expressed as a number or a vector. These values or vectors are used to represent these various kinds of pixel point sets in order to make it easier for the computer to comprehend them. Features are a necessary component of any computer classification method. For various pictures, classification algorithms, and classification purposes, the features that need to be extracted are often different. In feature extraction, people tend to extract too many features. This will result in an increase in computations and superfluous characteristics, which will have a detrimental effect on categorization. As a consequence, the final classification outcome will be influenced by the quantity and efficiency of feature extraction and make a significant contribution. They prefer to use basic and refined characteristics for categories that are not as complex. There is a clear contrast in the gray level between the lesion and the surrounding normal tissue, as seen in the multiband picture above. Because the lesion region appears darker, the average gray value of the sample area was used as the first feature to be retrieved in this study. As for the classification algorithm, due to the small number of features, this paper uses the more commonly used *K*-means clustering algorithm to classify the surface of the cervical tissue.

Since the system is based on a combination of both the local area network and the Internet, the internal systems use the local area network for data exchange, and the system and users use the Internet for information transmission. As a result, inside the LAN, it is preferable to utilise a star topology logic structure (as illustrated in Figure 7). The reason is that the star topology logical structure is an online structure in which the server (switch) is the centre, and all computers are connected to the server (switch). This structure can prevent each computer from affecting each other when a failure occurs and can work independently, and the real wiring of this star-shaped structure will not be very difficult, as long as there is enough connection medium.

In terms of connection of form data, the connection between forms can be divided into two types. One is to use ADODC, the most common connection method for forms, which is the connection method used for form connection. The page link is generated using a relative route as a hyperlink in this method. As long as the link target file exists in the folder, the hyperlink may be generated using this method without thinking about the computer's path. As a result, when the location of the system folder changes, the hyperlink route does not have to be adjusted. Using data transfer between dynamic web pages as a connection mechanism. Programming is used to make this happen. The linking method can be based on the needs of the editor, what data and how much data is sent to that page, and what operations are performed on the data. In fact, this kind of link is a way of linking data. The difficulty of this link method is that because it is derived from programming, the correctness of the compiled program must be ensured. If the correctness is not ensured, the link to the web page will not work correctly.

The manual module process in this system includes evaluation of fresh image information, change of picture information, and review after picture processing, as illustrated in Figure 8.

After constructing the above system model, the performance of the system is verified, and the intelligent diagnosis effect of cervical cancer is evaluated based on the actual situation. This article primarily performs research from three aspects in the system evaluation: picture feature identification, diagnostic and treatment accuracy, and user experience. The results are shown in Table 1 and Figure 9.

From the above research, the cervical cancer intelligent diagnosis system based on the data mining algorithm proposed in this paper has a good auxiliary diagnosis effect, which can be verified in clinical practice in the follow-up.

## 5. Conclusion

With the advancement of information technology, computer systems have been more widely utilised in the service sector, particularly in hospitals. The Gynecology Research Office of the hospital is mainly responsible for judging the pictures of cervical cancer cells, classifying the results of judging cells, and judging diseased cancer cells, normal cells, and suspected cells. However, these operations must rely on image processing software for processing. For front and back ends, the data centre uses database software and system development tools to actualize them. The business processing centre will be kept in a different environment. To avoid severe mistakes due to catastrophic failures, the business and data processing environment is protected in this way. Use of image data to segment cervical cancer cell images, picking feature vectors based on cell characteristic information, and development of a classifier using statistical methods are all discussed in this article. According to the results of the tests, this system has a strong automatic recognition effect and a good supplementary diagnostic effect. Therefore, clinical practice in follow-up may verify it.

## Figures and Tables

**Figure 1:** The process of processing cervical cancer diagnosis and classification problems.

**Figure 2:** Flow chart of discretization of continuous attributes for cervical cancer intelligent diagnosis.

**Figure 3:** Frame structure of the automatic analysis system for cervical cancer cell images.

**Figure 4:** Flow chart of image registration.

**Figure 5:** Bilinear interpolation.

**Figure 6:** The flow of the optimized auxiliary diagnosis algorithm.

**Figure 7:** Topology diagram of cervical cancer intelligent diagnosis system based on data mining.

**Figure 8:** The new organizational structure chart.

**Figure 9:** Statistics of system performance test results.

**Table 1:** Statistics of intelligent diagnosis results of cervical cancer based on data mining.

Number	Feature recognition	Accuracy	User experience
1	94.64	84.72	91.91
2	93.70	89.08	88.23
3	96.57	86.50	84.39
4	91.80	85.41	80.05
5	94.84	85.67	93.58
6	91.73	86.45	94.04
7	92.12	87.17	83.04
8	95.34	87.64	90.59

## Data Availability

The data used to support the findings of this study are included within the article.
